# Expression and significance of NELIN and SM22α in varicose vein tissue

**DOI:** 10.3892/etm.2015.2170

**Published:** 2015-01-08

**Authors:** SHIHUI CHEN, SHIYONG QIN, MINGHAI WANG, SHUGUANG ZHANG

**Affiliations:** 1 Department of Vascular Surgery, Dezhou Municipal Hospital, Dezhou, Shandong 253000, P.R. China; 2 Department of Vascular Surgery, Qianfoshan Hospital Affiliated to Shandong University, Jinan, Shandong 250014, P.R. China

**Keywords:** varicose veins, NELIN, SM22α, phenotypic transition, vascular smooth muscle cell

## Abstract

The aim of the present study was to investigate the expression of NELIN and SM22α in lower extremity varicose vein tissue, and their association with varicose veins. Tissue samples were collected from 18 patients with lower extremity varicose veins for the experimental group, while normal great saphenous vein tissue was reserved during coronary artery bypass surgery from 14 patients for the controls. Reverse transcription polymerase chain reaction (RT-PCR) analysis was applied to detect the mRNA expression levels of NELIN and SM22α, while immunohistochemical techniques were used to detect the protein expression levels in the normal and abnormal veins. RT-PCR results revealed that the mRNA expression levels of NELIN and SM22α in the experimental group decreased significantly when compared with the control group (P<0.01). In the two groups, immunohistochemical staining demonstrated that NELIN and SM22α were primarily expressed in the cytoplasm of smooth muscle cells, and the expression quantity decreased significantly in the experimental group when compared with the control group (P<0.05). The low expression of SM22α in the primary lower limb varicose vein tissue indicated that the vascular smooth muscle cell layer had transformed from a contractile to a secretory phenotype, which may have resulted in the remodeling of the vein walls and the occurrence of varicose veins. Therefore, NELIN and SM22α were demonstrated to play a key role in the development of varicosity.

## Introduction

Vascular smooth muscle cells (VSMCs) are a highly specialized type of cell, whose primary functions in mature animals include contraction (1) and the production of matrix components of the blood vessel wall (2). The proliferation of VSMCs has been demonstrated to be important in the development of atherosclerosis (3). Fully differentiated or mature smooth muscle cells (SMCs) express a unique repertoire of contractile proteins, ion channels and signaling molecules that are required for functionality.

VSMCs exhibit a variety of phenotypes at different developmental stages, under different pathophysiological conditions or normal conditions, depending on the anatomical location of the vessels (4). Previous studies have aimed to distinguish between the two phenotypes of VSMCs, the spindle-shaped ‘contractile’ and epithelioid-shaped ‘synthetic’ phenotypes (5). Varicose veins exhibit thickened vessel walls, as a result of the dysregulation of the synthesis of extracellular matrix proteins in SMCs (6). The phenotypic modulation of SMCs can alter extracellular matrix metabolism (7), and the etiology and physiopathology of varicose disorders include venous wall remodeling associated with abnormalities of SMCs and extracellular matrix (8).

NELIN is a novel F-actin-associated protein that has been shown to have restricted expression in the heart, skeletal muscle, arteries and veins (9). The protein mediates cell motility and is important in the process of cell migration and adhesion (10). SM22α is a calponin-related protein (11) and one of the earliest markers of differentiated SMCs (12). The 6.2-kilobase single copy gene is composed of five exons, and is expressed in the smooth, cardiac and skeletal muscle lineages during early embryogenesis, prior to becoming restricted specifically to VSMCs during late fetal development and adulthood (13).

The mechanisms and determinants underlying the development of varicosities are not yet clearly defined. In the present study, the transcriptional and translational expression levels of NELIN and SM22α in varicose vein and normal vein tissues were analyzed. The aims of the study were to verify the phenotypic modulation of VSMCs in varicose vein tissues, and discuss the possible mechanisms underlying the development of varicose veins.

## Materials and methods

### Specimen collection

In total, 18 patients with lower limb varicose veins, who had undergone treatment at the Qianfoshan Hospital Affiliated to Shandong University (Jinan, China), were assigned to the experimental group. The average age of the patients was 46.6±15.5 years, and 10 patients were male. In addition, 14 patients that had undergone great saphenous vein coronary artery bypass surgery were assigned to the control group. These patients had an average age of 46±13 years, and five patients were female. The patients in the control group did not have a medical history of varicose veins, which was verified by various preoperative assessments. During surgery, tissue samples from the great saphenous vein were obtained from the two groups, with two samples collected for each case. One sample was quick-frozen and immediately stored in a liquid nitrogen container, while the other sample was soaked in 10% formaldehyde solution to be fixed for 24 h, then conventionally dehydrated, hyalinized, embedded in wax and cut into 4-μm slices for preservation. Written informed consent was provided by the patients, and sample and data collection were approved by the Ethics Committee of Qianfoshan Hospital Affiliated to Shandong University.

### Main reagents

TransZol Up and two-step reverse transcription polymerase chain reaction (RT-PCR) kits were purchased from Beijing TransGen Biotech Co., Ltd. (Beijing, China). β-actin upstream and downstream primers were synthesized by Takara Bio, Inc. (Shiga, Japan). NELIN-specific, SM22α-specific and GAPDH upstream and downstream PCR primers were synthesized by Beijing Dingguo Changsheng Biotechnology Co., Ltd. (Beijing, China). A rabbit anti-human anti-NELIN polyclonal antibody was purchased from Sigma-Aldrich (St. Louis, MO, USA), while a concentrated rat anti-human SM22α polyclonal antibody was purchased from Proteintech Group, Inc. (Chicago, IL, USA). Two resistant kits for immunohistochemical streptavidin-biotin complex (SABC) detection were purchased from Wuhan Boster Biotechnology Co., Ltd. (Wuhan, China). Diaminobenzidine (DAB) staining reagents were purchased from Beijing Zhongshan Jinqiao Biotechnology Co., Ltd. (Beijing, China), and all other reagents were homebred and analytically pure.

### RT-PCR detection of NELIN and SM22α mRNA expression in the vein tissue

Total RNA in the vein tissue was extracted with TransZol Up, and the purity of the RNA samples was determined by an ultraviolet (UV) spectrophotometer (EU-2800; Shanghai Onlab Instruments Co., Ltd., Shanghai, China). The specific PCR primer sequences of human β-actin and NELIN are shown in Table I, while the sequences of GAPDH and SM22α are shown in Table II. The synthesis of first-strand cDNA and PCR were conducted according to the manufacturer’s instructions of the two-step RT-PCR kit. The RT-PCR for NELIN included 2X Easy*Taq* PCR SuperMix (25 μl), cDNA (10 μl), upstream and downstream primers of NELIN (1.0 μl each), upstream and downstream primers of β-actin (1.0 μl each) and double-distilled (dd) H_2_0 (11 μl). The thermal cycle format used in the RT-PCR was as follows: One cycle of preheating at 94°C for 2 min; 31 amplified cycles with denaturation for 30 sec at 94°C, annealing for 30 sec at 55°C and extension for 45 sec at 72°C; followed by a final incubation cycle at 72°C for 10 min. The RT-PCR for SM22α PCR included cDNA (2 μl), upstream and downstream primers of SM22α (0.5 μl each), upstream and downstream primers of GAPDH (0.5 μl each), 2X Trans*Taq*™ High Fidelity PCR SuperMix II (25 μl) and ddH_2_0 (21 μl). The thermal cycle format used in the RT-PCR was as follows: 33 cycles of denaturation for 30 sec at 94°C, annealing for 30 sec at 56°C and extension for 30 sec at 72°C; followed by a final incubation cycle at 72°C for 10 min. Products of 10 μl (each) were analyzed by electrophoresis in 1.5% agarose gels and visualized under UV illumination. The products were photographed using an independent softwae package controlled by a gel imaging system (GelDol2000; Bio-Rad, Hercules, CA, USA) and semi-quantified with density scanning. The objective stripe and internal control products were compared. The ratio of the density scanning values of NELIN against the GAPDH control was used to evaluate the expression level of NELIN mRNA. To analyze the differences between the experimental and control groups, the mRNA expression level of SM22α was evaluated by comparing the ratio of the density scanning values of SM22α against the GAPDH control.

### SABC immunohistochemistry staining

Tissue samples were cut into slices, dewaxed and immersed in water. Endogenous peroxide was blocked by incubating the tissues with 3% H_2_O_2_, after which antigen retrieval (hot repair with microwave) was conducted. Tissues were blocked with 5% bovine serum albumin, and incubated with primary antibodies against NELIN (rabbit anti-human, 1:150) and SM22α (polyclonal, 1:100) for 60 min at room temperature. Subsequently, the samples were incubated with a secondary antibody for 20 min, which was followed by the addition of the avidin-biotin peroxidase complex. Staining was visualized with DAB and tissues were counterstained with hematoxylin solution, then for transparent and sealed in piece with neutral gum. At every stage of the dyeing process, phosphate-buffered saline was used to replace the primary antibodies as the negative control.

Under a light microscope (BX-51; Olympus Corporation, Center Valley, PA, USA), positive staining (yellow or brown-yellow) was observed in the cytoplasm of the VSMCs. For image analysis, five evenly dyed and completely non-overlapping outlines were selected from each slice to be photographed under 10×40 magnification; all the images were exactly the same size. Integral optical density (IOD) values of each image were determined using Image-Pro Plus 5.0 image analysis software (Media Cybernetics, Rockville, MD, USA) and the average value was calculated. A positive correlation was observed between the IOD value and the protein expression of positive cells; this value was regarded as the semi-quantitative value of the sample.

### Statistical analysis

Results are expressed as the mean ± standard deviation. Mean values were compared by analysis of variance with the Student-Newman Keuls test, using SPSS 10.0 software (SPSS, Inc., Chicago, IL, USA). P<0.05 was considered to indicate a statistically significant difference.

## Results

### RT-PCR

RT-PCR analysis revealed that the mRNA expression levels of NELIN in the VSMCs were significantly decreased in the experimental group (0.2867±0.1025) when compared with the control group (0.4221±0.220; P<0.01; Fig. 1). Similarly, the mRNA expression levels of SM22α were significantly reduced in the experimental group (0.2614±0.1168) when compared with the control group (0.5114±0.1554; P<0.01; Fig. 2).

### SABC immunohistochemistry

Positive staining of NELIN (Fig. 3) and SM22α (Fig. 4) was observed in the cytoplasm of the cells. Immunohistochemical staining revealed a significant decrease in the expression levels of NELIN and SM22α in the experimental group when compared with the control (P<0.05). According to the statistical analysis, the IOD value of the NELIN protein staining was significantly reduced in the experimental group (7422.56±2423) when compared with the control group (9785.85±3005.85; P<0.05; Fig. 5). Similarly, the IOD value of SM22α staining was significantly reduced in the experimental group (10054.79±3584.07) when compared with the control group (16226.05±3378.16; P<0.05; Fig. 6).

## Discussion

As shown in a previous study, VSMCs cultivated *in vitro* change from a contractile to a synthetic phenotype following four subcultures, with the symbol of phenotypic transition being a clear reduction in SM22α expression in the VSMCs (14). Therefore, in the present study, the expression of SM22α was analyzed to assess the occurrence of VSMC phenotypic transition in the varicose vein tissues. The results revealed that the VSMCs in the control group were primarily of a contractile phenotype (15), while in the control group, a number of VSMCs had changed from a contractile to a synthetic phenotype (16). This result was consistent with previous study of VSMC *in vitro* culturing. The increase in synthetic phenotype VSMCs may result in an increase in extracellular matrix immaturity, resulting in a decrease in the normal extracellular matrix maintenance of cell stability and wall integrity. Subsequently, structural changes may occur in the normal vein tissues, which can be verified by the morphological differences of the two groups of specimens observed under immunohistochemical light and electron microscopy. Based on the phenotypic transition, the vein wall structure changes and causes venous dilation (17). An increase in the vein wall tension augments the expression/activity of matrix metalloproteinases, which induces the degradation of the extracellular matrix proteins and affects the structural integrity of the vein wall, ultimately leading to chronic and progressive venous insufficiency and varicose vein formation (18).

NELIN expression was observed in the VSMCs of the vein wall; however, the mRNA and protein expression levels were markedly reduced in the lower limb varicose vein tissue. These results indicated that the downregulation of NELIN expression may be a branch sign of VSMC phenotypic transition. A previous study reported that NELIN was a novel F-actin-binding protein that was colocalized with F-actin and filamin in the cytoplasm of cells (19). Therefore, NELIN was hypothesized to be associated with the skeleton organization of VSMCs, regulating a variety of biological behaviors, including the phenotype, form and systolic function of the cytoskeleton, directly or indirectly.

Sequence analysis has previously indicated that amino acids 154–161 of SM22α may be an actin-binding site (20). In addition, amino acids 175–195 have been shown to exhibit a high homology with tandem repeat domains in the COOH-terminal of calponin h1 and h2; in calponin, these tandem repeat sequences are important for full actin affinity (21). NELIN and SM22α were hypothesized to combine with actin simultaneously, resulting in a change of form and function of the cytoskeleton. A cell phenotypic transition may subsequently occur, promoting the occurrence of varicose veins.

In conclusion, the present study demonstrated that VSMCs in varicose vein tissue transformed from a contractile to a synthetic phenotype with varicosity. Furthermore, NELIN and SM22α are important for the phenotypic transition. Since NELIN and SM22α are actin-binding proteins, a synergistic effect may exist between them. However, the specific regulatory and molecular mechanisms underlying the mutual coordination remain unclear and require further study.

## Figures and Tables

**Figure 1:** Reverse transcription polymerase chain reaction analysis revealed weak mRNA expression of NELIN in the vascular smooth muscle cells (VSMCs) of the experimental group, but strong expression in the control group. (A) Expected length of the PCR products was 611 bp (NELIN) and 312 bp (β-actin). Lanes: N, control group; X, DNA marker DL 2000; and P, experimental group. (B) Downregulation of NELIN mRNA expression in the VSMCs from the varicose vein tissue. Data are presented as the mean ± standard deviation.

**Figure 2:** Reverse transcription polymerase chain reaction analysis revealed weak mRNA expression of SM22α in the vascular smooth muscle cells (VSMCs) of the experimental group, but strong expression in the control group. (A) Expected length of the PCR products was 232 bp (SM22α) and 472 bp (GADPH). Lanes: N, control group; X, DNA marker DL 2000; and P, experimental group. (B) Downregulation of SM22α mRNA expression in the VSMCs from the varicose vein tissue. Data are presented as the mean ± standard deviation.

**Figure 3:** Immunohistochemical staining revealed NELIN expression in the cytoplasm of the (A) experimental and (B) control groups.

**Figure 4:** Immunohistochemical staining revealed SM22α expression in the cytoplasm of the (A) experimental and (B) control groups.

**Figure 5:** IOD of NELIN protein expression staining. Vascular endothelial growth factor expression was significantly decreased in the experimental group compared with the control group (P<0.05). Data are presented as the mean ± standard deviation. IOD, integral optical density.

**Figure 6:** IOD of SM22α protein expression staining. Vascular endothelial growth factor expression was significantly decreased in the experimental group compared with the control group (P<0.05). Data are presented as the mean ± standard deviation. IOD, integral optical density.

**Table I:** Primer sequences used for reverse transcription polymerase chain reaction analysis of NELIN.

Gene	Primer	Amplified fragment length (bp)
NELIN		
Positive-strand	5′-AGGAGTGGCTCTATTCAA-3′	611
Negative-strand	5′-GGTAAGTAAAGGCAGTAAG-3′	
β-actin		
Positive-strand	5′-TTCTGTGGCATCCACGAAACT-3′	312
Negative-strand	5′-TTCTGTGGCATCCACGAAACT-3′	

**Table II:** Primer sequences used for reverse transcription polymerase chain reaction analysis of SM22α.

Gene	Primer	Amplified fragment length (bp)
SM22α		
Positive-strand	5′-TGGTGAACAGCCTGTACCCT-3′	235
Negative-strand	5′-CACGGTAGTGCCCATCATTC-3′	
β-actin		
Positive-strand	5′-ACCACAGTCCATGCCATCAC-3′	472
Negative-strand	5′-TCCACCACCCTGTTGCTGTA-3′	
